The article "Severe headache as a key symptom in bilateral idiopathic adrenal hyperplasia-induced primary hyperaldosteronism: A case report" was retracted in 2025. Reasons: unreliable results or conclusions; concerns about the authorship; concerns about the article.

# Severe headache as a key symptom in bilateral idiopathic adrenal hyperplasia-induced primary hyperaldosteronism: A case report

**DOI:** 10.1097/MD.0000000000042164

**Published:** 2025-04-18

**Authors:** Ali Safaa Abduljabbar, Hashim Talib Hashim, Ahmed Dheyaa Al-Obaidi, Ashraf Fhed Mohammed Basalilah, Israa Al-gburi, Zaid Saad Abed Madhi

**Affiliations:** a University of Baghdad, College of Medicine, Baghdad, Iraq; b University of Warith Al-Anbiyaa, College of Medicine, Karbala, Iraq; c Hadhramaut Hospital, Hadhramaut, Yemen; d Indiana University, School of Medicine, Indianapolis, IN; e Radiology Techniques Department, College of Health and Medical Techniques, Al-Mustaqbal University, Babylon, Iraq.

**Keywords:** adrenal hyperplasia diagnosis, bilateral idiopathic adrenal hyperplasia, endocrine hypertension, headache, hyperaldosteronism, hypertension

## Abstract

**Rationale:**

Severe headaches can have various causes, but they are commonly associated with common conditions such as tension-type headaches or migraines. However, in cases where these common causes do not explain the symptoms, it becomes essential to investigate secondary causes. This case highlights the importance of considering rare conditions, such as bilateral idiopathic adrenal hyperplasia-induced primary hyperaldosteronism, as a potential cause of persistent headaches and refractory hypertension. The study aims to explore the relationship between primary hyperaldosteronism and severe headaches, emphasizing the importance of early diagnosis and appropriate treatment for improving patient outcomes.

**Patient concerns:**

A 25-year-old male presented with severe, sporadic occipital headaches that had been ongoing for 2 months.

**Diagnoses:**

Initial tests, including a complete blood count, thyroid-stimulating hormone levels, and echocardiography were normal. Despite antihypertensive treatment, his blood pressure remained elevated. Further investigations revealed a high aldosterone-to-renin ratio, indicative of primary hyperaldosteronism. Imaging confirmed the diagnosis of bilateral idiopathic adrenal hyperplasia.

**Treatment:**

Management of bilateral idiopathic adrenal hyperplasia involves medical therapy with mineralocorticoid receptor antagonists like spironolactone or eplerenone. These medications block the effects of aldosterone, helping to control blood pressure and correct electrolyte imbalances.

**Outcomes:**

The patient’s refractory hypertension to initial therapies underscores the necessity of considering secondary causes of hypertension early in the diagnostic process, particularly in young patients without a significant family history of hypertension.

**Lessons:**

This case highlights the importance of considering secondary causes of hypertension and severe headaches when common treatments do not yield the expected results. Timely diagnosis of conditions like primary hyperaldosteronism can significantly improve patient outcomes through targeted therapy.

The article "Severe headache as a key symptom in bilateral idiopathic adrenal hyperplasia-induced primary hyperaldosteronism: A case report" was retracted in 2025. Reasons: unreliable results or conclusions; concerns about the authorship; concerns about the article.

## 1. Introduction

Severe headaches are a prevalent clinical complaint, often challenging to diagnose due to their multifaceted etiology.^[1]^ Common causes range from tension-type headaches and migraines to more serious conditions such as vascular disorders and intracranial pathologies. Understanding the underlying cause of severe headaches is crucial for effective treatment and management. When patients present with refractory symptoms despite standard treatments, it prompts healthcare providers to delve deeper into potential secondary causes, including endocrine disorders. Hypertension, commonly associated with severe headaches, requires careful evaluation, especially when it is resistant to conventional antihypertensive therapies.^[2]^ In rare instances, conditions like primary hyperaldosteronism, particularly due to bilateral idiopathic adrenal hyperplasia, might be the underlying cause. This case underscores the need for thorough investigation when faced with atypical presentations of common symptoms.^[3]^

## 2. Case presentation

A 25-year-old male sales distributor presented with sporadic episodes of moderate to sever headaches, mainly located in the occipital area. The onset of these headaches occurred 2 months ago, with each episode lasting anywhere from a few hours to 5 days. The headaches were characterized by tension-like pain and did not radiate. There were no additional symptoms present, such as weakness in the limbs, abnormal body movements, difficulties with speech, or altered mental state. In addition, the headaches were not accompanied with photophobia, phonophobia, nausea, or vomiting. Blood pressure measurements taken at home were high, averaging 190/100 mm Hg, but he did not seek medical attention instantly. Over the course of a week, he recorded his blood pressure 3 times a day and averaged 180/110.

At the first clinical visit, a complete blood count, urea and electrolytes, urine analysis, thyroid-stimulating hormone, electrocardiogram, and echocardiography were all performed, and the results were normal. He was prescribed an angiotensin II receptor blocker and later other drugs, but his blood pressure remained elevated, averaging 170/100 mm Hg. Upon presenting the clinic 7 weeks after initiating treatment, a thorough evaluation of the patient’s medical history was conducted. The patient denied experiencing any other neurological symptoms except from the occipital headache. The patient did not experience any chest pain, palpitations, difficulty breathing, fainting, or swelling in the ankles. No symptoms of hyperthyroidism, acromegaly, Cushing syndrome, or pheochromocytoma were observed. In addition, he did not exhibit any symptoms of oliguria, hematuria, or polyuria. His medical and surgical history did not show any significant events, and there was no history of hypertension in his family at a young age. He had recently used irbesartan for a period of 2 weeks, followed by a combination of irbesartan and hydrochlorothiazide for 3 weeks. He then switched to telmisartan/amlodipine for 2 weeks before presenting to clinic. The patient had a notable smoking history, smoking 1.5 packs of cigarettes daily for a duration of 7 years, resulting in a total of 10.5 pack-years.

The article "Severe headache as a key symptom in bilateral idiopathic adrenal hyperplasia-induced primary hyperaldosteronism: A case report" was retracted in 2025. Reasons: unreliable results or conclusions; concerns about the authorship; concerns about the article.

Upon examination, the patient had an average body build. His heart rate was 80 beats per minute, with a normal rhythm, volume, and character. The blood pressure was 170/100 mm Hg on both sides. The oxygen saturation level in the ambient air was 97%. There was no indication of Cushing syndrome, hyperthyroidism, or acromegaly. The cardiorespiratory evaluation was normal, and no renal artery bruit was detected.

He was sent for further investigations which revealed a serum potassium was 3.6 mEq/L (normal: 3.5–5.0 mEq/L) despite being on telmisartan; hemoglobin level was 16 g/dL (normal: 13.8–17.2 g/dL); white blood cell count was 8.4 × 10^3^/µL (normal: 4.5–11.0 × 10^3^/µL); platelet count was 267 × 10^3^/µL (normal: 150–450 × 10^3^/µL); blood urea level was 21 mg/dL (normal: 15–45 mg/dL); serum creatinine was 0.6 mg/dL (normal: 0.6–1.2 mg/dL); urine analysis showed no proteinuria; thyroid-stimulating hormone was 2.7 mIU/L (normal: 0.4–4.0 mIU/L); LDL cholesterol was 106 mg/dL (normal: <100 mg/dL desirable); HDL cholesterol was 45 mg/dL (normal: >40 mg/dL for men); triglyceride level was 190 mg/dL (normal: <150 mg/dL). Renal ultrasound and Doppler of renal arteries were normal. Plasma aldosterone was 31.2 µg/dL (normal: <16 µg/dL in a seated position); plasma renin activity was 1.1 ng/mL/h (normal: 1.0–2.6 ng/mL/h in a seated position); and the aldosterone-to-renin ratio was 28.36 (normal: <20). The patient was scheduled for a saline suppression test, but due to financial constraints, a CT adrenal protocol was performed instead, which indicated bilateral borderline thickness of the limbs of the adrenal glands maximally seen at the left posterior limb measuring 4.5 mm and at right posterior limb measuring 4.2 mm (Fig. 1). The final diagnosis was primary hyperaldosteronism due to bilateral idiopathic adrenal hyperplasia. He was started on spironolactone with titration of dosage while continuing taking telmisartan/amlodipine. After 2 weeks, his average blood pressure dropped to 140/85 mm Hg and then to 135/80 mm Hg a week later. Following the commencement of the new treatment regimen, the headaches resolved within 5 days.

The article "Severe headache as a key symptom in bilateral idiopathic adrenal hyperplasia-induced primary hyperaldosteronism: A case report" was retracted in 2025. Reasons: unreliable results or conclusions; concerns about the authorship; concerns about the article.

**Figure 1.** An enhanced CT scan of the abdomen for showing bilateral borderline thickness of the limbs of the adrenal glands.

### Outcomes

The patient demonstrated a significant reduction in blood pressure after the commencement of spironolactone therapy, leading to symptom resolution. The blood pressure decreased from 170/100 to 135/80 mm Hg over the course of a few weeks. The occipital headaches that had persisted for months resolved within 5 days of the treatment, highlighting the positive outcome of managing the underlying cause of hypertension and headaches.

## 3. Discussion

The case of a young male with severe headaches and persistent hypertension despite standard antihypertensive treatment led to a diagnosis of bilateral idiopathic adrenal hyperplasia-induced primary hyperaldosteronism. This diagnosis was confirmed through biochemical testing showing an elevated aldosterone-to-renin ratio and imaging studies.^[4]^

Primary hyperaldosteronism (PHA) is characterized by excessive production of aldosterone, leading to sodium retention, potassium excretion, and hypertension. It can be caused by unilateral adrenal adenoma, bilateral adrenal hyperplasia, or, less commonly, adrenal carcinoma. In this case, bilateral adrenal hyperplasia was identified, a less frequent but significant cause of PHA.^[5,6]^

The clinical presentation of PHA can vary. While hypertension is a hallmark, the presence of severe headaches, as in this case, emphasizes the broader symptomatology that can accompany this condition. Patients often present with nonspecific symptoms that can easily be attributed to more common conditions. This can delay the diagnosis, as seen with the patient’s initial management focusing on primary headache disorders and essential hypertension.^[7,8]^

Endocrine evaluations, including measurement of serum aldosterone, plasma renin activity, and subsequent aldosterone-to-renin ratio, are pivotal in diagnosing PHA. In this patient, the ratio was significantly elevated, suggesting autonomous aldosterone production. Imaging studies, such as CT or MRI of the adrenal glands, further aid in differentiating between unilateral and bilateral disease, guiding treatment decisions.^[9,10]^

Management of bilateral idiopathic adrenal hyperplasia involves medical therapy with mineralocorticoid receptor antagonists like spironolactone or eplerenone. These medications block the effects of aldosterone, helping to control blood pressure and correct electrolyte imbalances. The patient’s refractory hypertension to initial therapies underscores the necessity of considering secondary causes of hypertension early in the diagnostic process, particularly in young patients without a significant family history of hypertension.^[11–13]^

The article "Severe headache as a key symptom in bilateral idiopathic adrenal hyperplasia-induced primary hyperaldosteronism: A case report" was retracted in 2025. Reasons: unreliable results or conclusions; concerns about the authorship; concerns about the article.

## 4. Conclusion

In conclusion, this case illustrates the importance of a comprehensive approach to diagnosing severe headaches and hypertension, especially when initial treatments are ineffective. Bilateral idiopathic adrenal hyperplasia-induced primary hyperaldosteronism, although rare, should be considered in the differential diagnosis. Timely identification and appropriate management of such endocrine disorders can prevent complications and improve patient outcomes. This case also highlights the need for increased awareness among clinicians regarding the diverse presentations of endocrine hypertension.

### Limitations

Although this study presents a rare case, it has limitations that should be acknowledged. One key limitation is the lack of long-term follow-up after the resolution of symptoms. Additionally, due to financial constraints, some diagnostic tests (e.g., saline suppression test) were not conducted, which may have affected the overall diagnostic certainty. Moreover, the sample size is limited to a single case, which may reduce the generalizability of the findings.

## Acknowledgments

We thank all the authors to participate in the study.

## Author contributions

**Conceptualization:** Ali Safaa Abduljabbar, Hashim Talib Hashim, Zaid Saad Abed Madhi.

**Data curation:** Ali Safaa Abduljabbar, Hashim Talib Hashim, Ashraf Fhed Mohammed Basalilah, Israa Al-gburi.

**Formal analysis:** Ahmed Dheyaa Al-Obaidi.

**Investigation:** Ahmed Dheyaa Al-Obaidi.

**Methodology:** Ahmed Dheyaa Al-Obaidi.

**Project administration:** Ashraf Fhed Mohammed Basalilah.

**Resources:** Hashim Talib Hashim, Ahmed Dheyaa Al-Obaidi, Ashraf Fhed Mohammed Basalilah.

**Software:** Ashraf Fhed Mohammed Basalilah.

**Supervision:** Ali Safaa Abduljabbar, Hashim Talib Hashim, Israa Al-gburi, Zaid Saad Abed Madhi.

**Validation:** Ali Safaa Abduljabbar, Israa Al-gburi.

**Visualization:** Israa Al-gburi.

**Writing – original draft:** Ali Safaa Abduljabbar, Hashim Talib Hashim.

**Writing – review & editing:** Ahmed Dheyaa Al-Obaidi, Ashraf Fhed Mohammed Basalilah, Zaid Saad Abed Madhi.
